The article "Intelligent Noise Reduction Algorithm to Evaluate the Correlation between Human Fat Deposits and Uterine Fibroids under Ultrasound Imaging" was retracted in 2023. Reasons: signs of a paper mill; suspected computer-generated content; unreliable results or conclusions; lack of ethics approval or compliance.

# Intelligent Noise Reduction Algorithm to Evaluate the Correlation between Human Fat Deposits and Uterine Fibroids under Ultrasound Imaging

**DOI:** 10.1155/2021/5390219

**Published:** 2021-11-30

**Authors:** Yan Luo, Wenxia Huang, Kewei Zeng, Chunfeng Zhang, Chunyan Yu, Wencui Wu

**Affiliations:** ^1^Department of Ultrasound, Affiliated Hospital of Zunyi Medical University, Zunyi 563000, Guizhou, China; ^2^Department of Ultrasound Medicine, Haikou Hospital of the Maternal and Child Health, Haikou 571100, Hainan, China

## Abstract

This study aimed to realize the automatic diagnosis of fatty degeneration of uterine fibroids. In this study, the traditional nonlocal means (NLM) algorithm was improved by changing the Euclidean distance and introducing a cosine function and applied to the ultrasonic imaging intelligent diagnosis of patients with fatty degeneration of uterine fibroids. Then, the noise reduction effect of the improved NLM algorithm was evaluated based on several indicators, such as peak signal-to-noise ratio (PSNR), mean square error (MSE), contrast-to-noise ratio (CNR), figure of merit (FOM), and structural similarity (SSIM). The accuracy, sensitivity, specificity, and *F*1 score were adopted to evaluate the improved NLM algorithm for diagnosing fatty degeneration of uterine fibroids, and the Perona–Malik (PM) algorithm and NLM algorithm were used for comparative analysis. The results showed that after the ultrasound images of patients with uterine fibroids were denoised using the improved NLM algorithm, the PSNR, MSE, CNR, FOM, and SSIM were obviously better than the same indicators of the image processed with the PM algorithm and the NLM algorithm, and the differences were statistically significant (*P* < 0.05). The diagnosis results of patients with fatty degeneration of uterine fibroids found that there was only one patient with missed diagnosis after the ultrasound image was processed with NLM algorithm, and there was no statistical difference between the improved NLM algorithm and the assisted diagnosis accuracy of the pathological examination results (*P* > 0.05). The average noise reduction time of the PM algorithm, NLM algorithm, and the improved NLM algorithm was 16.38 ± 4.33 s, 18.01 ± 5.14 s, and 23.81 ± 4.62 s, respectively. The diagnosis rate before improvement was 75.0%, the diagnosis accuracy rate for PM was 79.69%, and that after improvement was 85.94%. In summary, the improved NLM algorithm showed a good noise reduction effect on ultrasound images of patients with uterine fibroids, could improve the diagnosis accuracy of fatty degeneration of uterine fibroids, and could assist clinicians in the ultrasound imaging diagnosis of patients with uterine fibroids.

## 1. Introduction

Uterine fibroid originates from uterine smooth muscle cells and is the most common benign tumor in the reproductive system of women of childbearing age [1]. Uterine fibroid is composed of smooth muscle and connective tissue. It is common in reproductive women between 30 and 50 years old. Clinical statistics show that the prevalence of uterine fibroid is about 20–40% in women of childbearing age and 51∼60% in women aged between 40 and 50 years, and its incidence has a trend of increasing year by year [2]. Fat deposits caused by obesity can cause metabolic disorders in various organs of the human body, and myocardial fatification leads to myocardial contraction and diastolic dysfunction [3, 4]. Excessive fat deposits will also be accompanied by obvious changes in the function of the nerve or endocrine system. In recent years, studies have found that obesity can increase the risk of uterine fibroids. Obesity may affect the development of uterine fibroids by changing the level of estrogen metabolism in women [5, 6].

Most patients with uterine fibroids have no obvious clinical symptoms, and they are often found occasionally during pelvic ultrasound examinations, so no treatment is usually required. Only about 20–50% of patients may have menstrual changes, chronic pelvic pain, lower abdomen masses, waist bulging, and compression symptoms. Uterine fibroid is currently one of the most common reasons for hysterectomy in menopausal women. However, hysterectomy changes the physiological status of women, causing great negative impacts on the physiology and physiology of patients and increasing the economic burden of patients and national economic expenditures [7]. If uterine fibroids are not treated in time, fat deformation will result. Fat deformation is a rare type of degeneration, accounting for about 0.2% of uterine fibroids. It usually occurs after necrosis or hyaline degeneration and often occurs in late hyalinosis or after necrosis. It may also be caused by fibroids mesenchymal metaplasia to form adipose tissue. The deformed lesions are relatively small and difficult to detect with the naked eye. There are also a small number of patients with some small fat particles, which are mainly manifested by the increase of fat particles in the cells of the fibroids. The muscle cells have vacuoles, and the fat staining is positive. When patients with uterine fibroids have steatosis, they should be treated according to their own symptoms in time to prevent the situation from getting worse and causing more damage to their health [8].

At present, there are two types of treatment for uterine fibroid: nonsurgical treatment and surgical treatment. Nonsurgical treatment includes drug treatment, conservative treatment, uterine artery embolization (UAE), high-intensity focused ultrasound (HIFU), and radiofrequency ablation (RFA) [9]. The choice of treatment for uterine fibroid depends largely on the clinical symptoms of the patient, but surgery is still the main treatment. Surgery is currently the most effective treatment method, including hysterectomy, laparoscopic myomectomy, hysteroscopic myomectomy, and open myomectomy, and it is the standard treatment of uterine fibroid, but it will cause some trauma to patients [10, 11].

Most uterine fibroids have obvious characteristics in the ultrasound image, which can be easily diagnosed by two-dimensional and color Doppler ultrasound. However, the diagnosis of some uterine fibroids is difficult due to their special location or complex image diagrams [12]. The incidence of uterine fibroid is about 0.4–0.8%, but the changes are diverse, including cystic degeneration, steatosis, hyaline degeneration, sarcomatoid degeneration, and erythroid degeneration. Uterine fibroids with and without fatty degeneration are clinically difficult to distinguish in terms of performance and the characteristics of the sonogram, and it is easy to cause missed diagnosis in the preoperative acoustic image diagnosis, so it mostly depends on the postoperative pathological examination [13, 14]. Fatty degeneration is a kind of very rare uterine fibroid, accounting for about 0.2% of the degeneration of uterine fibroids. The lesion of fatty degeneration is usually small and difficult to detect with the naked eye. Fatty degeneration of uterine fibroids is similar to the clinical manifestations of lipomas. It is impossible to make a clear diagnosis before surgery, which can easily lead to missed diagnosis and misdiagnosis [15]. At present, the preferred method for diagnosing fatty degeneration of uterine fibroid is ultrasonography. Two-dimensional ultrasonography of uterine fibroid without degeneration shows that the image is round or elliptical with clear boundaries. Semicircular or ring-shaped color blood flow signals can be seen under color Doppler ultrasound [16]. Undenatured uterine fibroids and fatty uterine fibroids show a different imaging morphology under ultrasound, so ultrasound diagnosis of uterine fibroids is of significant value. However, ultrasonic diagnosis of fatty degeneration of uterine fibroids can show complex sound and image characteristics and is affected by ultrasonic detection technology and its imaging mechanism. Due to the mutual interference of a large number of ion beams and the scattering and superposition of echo signals, noise will inevitably be generated, and noise will appear to a certain extent, which affects the observation of clinicians to the medical images and even lead to misdiagnosis of diseases [17]. Nonlocal Means Filtering (NLM) is an improved filtering algorithm proposed by Buades et al. based on the traditional neighborhood filtering method. NLM can make use of the self-similar nature of the image and make full use of the redundant information in the image. While denoising, it can keep the details of the image to the greatest extent. The similarity among all pixels in the image and the current pixel is calculated. Taking into account the amount of calculation and efficiency, two windows of fixed size are generally set. A large search window and a small neighborhood window, the neighborhood window slides in the search window, the influence of the corresponding center pixel on the current pixel is determined according to the similarity between the neighborhoods, and the image with a very good pixel can be outputted. Therefore, based on the ultrasound image noise reduction algorithm, the ultrasound images of patients with fatty degeneration of uterine fibroids were denoised intelligently. This study applied the NLM algorithm to ultrasound images to clearly and accurately present ultrasound images, to provide a basis for the ultrasound image noise reduction and imaging information analysis of patients with uterine fibroids and a theoretical basis for the clinical diagnosis of uterine fibroids.

## 2. Materials and Methods

### 2.1. Ultrasound Image Noise Reduction Method Based on Improved NLM Algorithm

Two-dimensional B-ultrasound was the main ultrasonic diagnostic technology in China. Ultrasound had various characteristics of sound waves. In the process of ultrasound propagation, ultrasound passed through tissues and organs with different structures, causing varying degrees of attenuation. The receiving end receives varying degrees of echoes, which were marked with light points of different gray levels on the screen to obtain the cut surface imaging of the tested organ or tissue [18]. Ultrasound underwent constructive interference and destructive interference during the return process. After being transformed into an image, speckle noise of varying brightness and darkness would appear on the image. In ultrasound imaging, the interference position of the ultrasound echo signal was random. Therefore, the speckle noise on the ultrasound image was also random [19]. In the resolution unit of the ultrasound image, a Rayleigh distributed random variable could be applied to describe the intensity of the ultrasound echo scattering signal. It is assumed that the scattering signal from each scattering point in the resolution unit was *M* and the phase offset was *θ*. Then, the superposition result could be expressed by the following equation:

(1) $$\begin{array}{c} M=Me^{\theta l}=\sum_{i=0}^{N-1}M_{i}e^{\theta_{i}l},\\ \xi_{i}=\frac{M_{i}}{\sqrt{N}}. \end{array}$$

It was assumed that the phase of the echo signal obeyed the normal distribution within [−*π*, *π*] and the number of scatterers in the resolution unit was large enough, the joint distribution of the real and imaginary parts was Gaussian, and the joint probability density could be expressed by the following equation:

(2) $$\begin{array}{c} P\left(M_{r},M_{i}\right)=\frac{1}{2\pi \sigma^{2}}\exp\left(-\frac{M_{r}^{2}+M_{i}^{2}}{2\sigma^{2}}\right). \end{array}$$

where *σ*^2^ represents the variance of the function, and the ultrasonic scattered wave signal can be expressed as the product of two Gaussian density functions, which could be shown as follows:

(3) $$\begin{array}{c} M=\sqrt{M_{r}^{2}+M_{i}^{2}}. \end{array}$$

The probability density function obtained by this is shown in the following:

(4) $$\begin{array}{c} \rho \left(M\right)=\left\{\begin{array}{cc} \frac{M}{\sigma^{2}}\exp\left(-\frac{M^{2}}{2\sigma^{2}}\right), & M\geq 0,\\ 0, & M<0. \end{array}\right. \end{array}$$

For noise reduction of the general image, logarithmic function transformation can be used to transform the system noise into additive noise, and finally, the inverse transformation could be performed. If *P*(*i*, *l*) represented a real noise-free image, *P′*(*i*, *l*) represented an input noise image, and *N*(*i*, *l*) referred to a multiplicative noise signal, the noise image contained *N*(*i*, *l*) can be expressed as follows:

(5) $$\begin{array}{c} P^{\prime }\left(i,l\right)=P\left(i,l\right)*N\left(i,l\right). \end{array}$$

The logarithms of both sides of (5) were taken synchronously, and the following equation could be obtained:

(6) $$\begin{array}{c} \ln\;P^{\prime }\left(i,l\right)=\ln\;P\left(i,l\right)*\;\ln\;N\left(i,l\right). \end{array}$$

When noise reduction was performed on a noisy image, it was easy to cause the destruction of the edge details of the image. An anisotropic diffusion filter model (PM model) could be introduced for processing, and its expression could be expressed as follows:

(7) $$\begin{array}{c} \frac{\partial I}{\partial t}=di\;v\left[c\left(\left|\nabla I\right|\right)\nabla I\right], \end{array}$$

(8) $$\begin{array}{c} I\left(t=0\right)=I_{0}. \end{array}$$

*I* represents the pixel to be processed, *div* represented the divergence operator, ∇ represents the gradient operator, and *t* refers to the number of iterations, which mean that the degree of noise reduction was related to the time or the number of iterations. According to the difference between the diffusion coefficient and the gradient, the following diffusion equation could be obtained:

(9) $$\begin{array}{c} c{\left(\left|\nabla I\right|\right)}_{1}=\frac{1}{1+{\left(\left|\nabla I\right|/k\right)}^{2}},\\ c{\left(\left|\nabla I\right|\right)}_{2}=\exp\left[-{\frac{\left|\nabla I\right|}{k}}^{2}\right]. \end{array}$$

The gradient amplitude in the PM model can detect the edge area of the image. When *c*(|∇*I*|) approached 0, the current pixel was the edge of the image, and the diffusion was suppressed; when *c*(|∇*I*|) approached 1, the diffusion was enhanced, and the discrete form of the PM model can be expressed as follows:

(10) $$\begin{array}{c} {\hat{I}}_{x}=I_{x}+\lambda \sum_{p\in N}c\left(\nabla I_{x,p}\right)\nabla I_{x,p}. \end{array}$$

In the equation above, *I*_*x*_ represents the discrete sampling of the noise image, *x* and *p* represent the pixel coordinates of the image, respectively, and *λ* represents the custom parameter for adjusting the degree of expansion. The PM algorithm could well retain the edge information of the image, but it was easily affected by the diffusion threshold during the noise reduction. When some isolated sharp noise points on the ultrasound image were processed, the gradient value was too large so that it was easy to be retained as the edge information of the image. When some image areas with little difference in gray level were filtered, it was easy to cause a block. Such noise removal method was based on the local mean of the noise image. It was easy to ignore the impact of sharp noise points when the noise of the image was reduced or removed. When the pixel gray value was replaced, some sharp noise points may be included in the image neighborhood to participate in the recalculation of the gray value of the central pixel, which in turn led to incomplete image noise reduction [20].

The NLM algorithm was originally a nonlocal image noise reduction algorithm based on the feature that the digital image contained a lot of redundant information. The NLM algorithm used all pixels in the image, so the noise reduction effect was better than the local average algorithm. The NLM algorithm took the pixel of the noisy image as the center, selected the appropriate neighborhood on the image, and then searched the entire image in the unit of the neighborhood pixel block. The possibility of noise contained in the pixel block with high similarity was lower, so a larger weight value could be assigned to the pixel block during the replacement. Conversely, the pixel block with lower similarity was more likely to contain noise, and it was difficult to represent the texture feature of the central pixel block, so the pixel block was assigned a smaller weight value.

For the pixels in a noisy image, the estimated pixel value calculated by the nonlocal mean algorithm can be expressed as follows:

(11) $$\begin{array}{c} \text{NL}\left(m\right)=\sum_{n}\varpi \left(m,n\right)v\left(n\right). \end{array}$$

where NL(*m*) is the pixel value calculated by the local average algorithm for the target pixel, *ϖ*(*m*, *n*) is the weight corresponding to the pixel *n*, and *v*(*n*) refers to the value of a certain pixel in other positions in the image. The similarity between *m* and *n* can be determined by the gray vectors *v*(*N*_*m*_) and *v*(*N*_*n*_). Then, the similarity between two gray levels can be expressed by the following equation:

(12) $$\begin{array}{c} \varpi \left(m,n\right)=\frac{1}{Z\left(m\right)}e^{{\left\|v\left(N_{m}\right)-v\left(N_{n}\right)\right\|}_{2,a}^{2}/h^{2}}. \end{array}$$

where *h* represents the filter coefficient, which controls the smoothness of the image. The smoother the image, the larger the *h*. In addition, *Z*(*m*) was defined as a normalized constant, and its function expression was written as follows:

(13) $$\begin{array}{c} Z\left(m\right)=\sum_{n}e^{{\left\|v\left(N_{m}\right)-v\left(N_{n}\right)\right\|}_{2,a}^{2}/h^{2}}. \end{array}$$

The NLM algorithm can make full use of the redundant information in the image to reduce noise while fully retaining the key information of the image. However, the time complexity of the NLM algorithm was high, there were still some artifacts in the denoised image, and there was a risk of image information loss when the image filter coefficient was large [21]. In the image processing of fatty degeneration of uterine fibroid patients, the difference in the spatial position of the edge of the lesion and the trunk of the blood vessel made it difficult for the similarity weight of the NLM algorithm to fully identify the similarity of the pixel blocks, leading to insufficient image noise reduction. Therefore, the NLM algorithm was improved. The traditional Euclidean distance is improved by using the block median value and the block average value and the gray value of the center pixel of the two pixel blocks, and the ratio of the three is improved to 2:3:2:

(14) $$\begin{array}{c} d=-\frac{1}{2}\left[2{\left(b\left(m\right)-b\left(n\right)\right)}^{2}+3{\left(a\left(m\right)-a\left(n\right)\right)}^{2}+2{\left(m-n\right)}^{2}\right]. \end{array}$$

where *b*(*m*) − *b*(*n*) represents the difference between the medians of pixel blocks *m* and *n*; *a*(*m*) − *a*(*n*) represents the difference between the means of pixel blocks *m* and *n*; and *m* − *n* represents the grayscale difference of the pixel block centered at *m* and *n*. In addition, the attenuation coefficient *h* can also measure the degree of image noise reduction, and its function expression can be expressed as follows:

(15) $$\begin{array}{c} h=\sqrt{2\beta \sigma \left|N\right|}. \end{array}$$

where *σ* represents the standard deviation, obtained directly by adding noise, but *σ* is unknown in the actual processing process. Therefore, the second method of noise variance estimation based on the Laplacian operator was adopted to adjust the added gradient value, and the improved noise variance could be calculated as follows:

(16) $$\begin{array}{c} \sigma^{\prime }=\sqrt{\frac{\pi }{2}}\frac{1}{6\left(W-2\right)\left(H-2\right)}\frac{\sum_{\forall m,n}\left|I\left(m,n\right)*M\right|\left|\nabla \right|}{\sum_{\forall m,n}\left|\nabla \right|},\\ \left|\nabla \right|=\frac{1}{1+{\left(2\left(\max\left|\nabla \right|\right)\right)}^{2}}. \end{array}$$

max|∇| represents the maximum gradient value in the horizontal and vertical directions of each pixel. The more complex the image texture structure, the larger the max|∇|. Based on (16), the gradient value can be reduced. Thereby, the overestimation of the noise variance could be weakened. The smoother the image texture area, the smaller the gradient value and the increase in the gradient weight. This method could effectively capture the noise signal on the image. At the same time, the cosine function was introduced to adjust the algorithm as a whole to make the gray transition of the image after noise reduction more balanced. The improved weight function expression is as follows:

(17) $$\begin{array}{c} w{\left(m,n\right)}^{\prime }=\exp\left(\frac{d}{2h^{2}}\right)\cos\left(\frac{\pi \;d}{2{\left(\left|N\right|+\left|H\right|\right)}^{2}}\right). \end{array}$$

Finally, the noise reduction processing of the entire noisy image was implemented in the search window, and the improved NLM image noise reduction algorithm is given as follows:

(18) $$\begin{array}{c} \text{NLM}\left[H\right]\left(m\right)=\frac{1}{\sum_{n\in H}w{\left(m,n\right)}^{\prime }}\sum_{n\in H}w{\left(m,n\right)}^{\prime }H\left(n\right). \end{array}$$

The algorithm combined the influence of the size of the search window on the effect of image noise reduction, adjusted the weight through the function *w*(*m*, *n*)′ to achieve a smooth transition of the overall gray value of the image, and made the noise reduction more thorough while preserving the basic details of the image. The calculating process of the improved NLM algorithm is shown in Figure 1.

### 2.2. Research Objects

In this study, 95 patients with fatty degeneration of uterine fibroids were selected as the research objects. All patients were treated at hospital from June 2019 to October 2020. All patients underwent postoperative pathological diagnosis and preoperative ultrasound diagnosis. The patients were 33∼69 years old, with an average age of 44.8 ± 9.36 years. All patients underwent total hysterectomy or myomectomy. During the surgery, the uterus of the patient was enlarged, the uterus morphology was normal, and nodule was seen on the endocervical wall, which was soft in quality with clear borders. This study had been approved by the Ethics Committee of hospital.

### 2.3. Ultrasound Diagnosis

All 95 patients who participated in this study underwent a color Doppler ultrasound diagnosis instrument (Color Doppler ultrasound instrument, DC-8PRO, Mindray) imaging examination, and the vaginal probe frequency was set to 6.0∼8.5 MHz. Before the examination, the patient was required to empty the bladder. The lithotomy position was selected, and the couplant was painted on the ultrasound probe, which was placed in the vaginal vault for examination. Firstly, the routine ultrasound was performed on the lesion of the patient to observe comprehensively by rotating the probe. The characteristics and size of the lesion were recorded. After the routine ultrasound examination, the lesion was examined with color Doppler to describe the blood supply of the lesion and determine related parameters. Finally, the entire uterine fibroid was performed with ultrasound imaging.

### 2.4. Evaluation of Noise Reduction Quality

The noise reduction effect was evaluated subjectively and objectively on the ultrasound images of all patients with uterine fibroids in this study. Subjective evaluation was mainly to evaluate the effect of image noise reduction through visual observation. It was easily affected by the subjective consciousness of the evaluator and lacked a quantitative standard to measure the quality of noise reduction effect. Therefore, some objective evaluation indicators were introduced for evaluation, including PSNR, MSE, CNR, FOM, and SSIM. They could be expressed as follows:

(19) $$\begin{array}{c} \mathrm{PSNR}=10\mathrm{lg}\left[\frac{pe_{\max}^{2}}{\left(1/h\cdot l\right)\sum_{a=1,b=1}^{h,l}{\left[f\left(a,b\right)-\hat{f}\left(a,b\right)\right]}^{2}}\right], \end{array}$$

(20) $$\begin{array}{c} \mathrm{MSE}=\frac{1}{h\cdot l}\sum_{a=1,b=1}^{h,l}{\left[f\left(a,b\right)-\hat{f}\left(a,b\right)\right]}^{2}, \end{array}$$

(21) $$\begin{array}{c} \mathrm{CNR}=\frac{2{\left(\mu_{a}-\mu_{b}\right)}^{2}}{\sigma_{a}^{2}+\sigma_{b}^{2}}, \end{array}$$

(22) $$\begin{array}{c} \mathrm{FOM}=\frac{1}{\max\left\{\hat{X},X_{\mathrm{ideal}}\right\}}\sum_{c=1}^{\hat{X}}\frac{1}{1+d_{c}^{2}\rho }, \end{array}$$

(23) $$\begin{array}{c} \mathrm{SSIM}\left(P,P^{\prime }\right)={\left[\mathrm{bri}\left(P,P^{\prime }\right)\right]}^{\alpha }\times {\left[\mathrm{con}\left(P,P^{\prime }\right)\right]}^{\beta }\times {\left[\mathrm{str}\left(P,P^{\prime }\right)\right]}^{\gamma }. \end{array}$$

where*pe*_max_ represents the maximum value of all pixels on the image; *h* and *l* refer to the height and width of the image, respectively; *f*(*a*, *b*) is the gray value of each pixel of the image without noise; $\hat{f}\left(a,b\right)$ stand for the gray value of each pixel of the image after noise reduction; Δ*f* and $\bar{\Delta }\overset{⌢}{f}$ represent the results of edge extraction of the original image *f* and the denoised image $\hat{f}$ by the 3 × 3 Laplacian operator, respectively; $\hat{X}$ is the number of boundary points after image processing; *X*_ideal_ means the number of ideal image boundary points; *d*_*c*_ represents the distance between the *c*^th^ boundary point and the closest boundary point after noise reduction; *P* and *P′* refer to the original ideal noise-free image and the noise-reduced image, respectively; and bri(*P*, *P*′), con(*P*, *P*′), and str(*P*, *P*′) refer to the brightness, contrast, and structure, respectively.

### 2.5. Evaluation of Diagnosis Accuracy

The accuracy, sensitivity, specificity, and *F*1 score were adopted to evaluate the prediction performance of the improved NLM algorithm, and the improved NLM algorithm was compared with the PM algorithm and NLM algorithm. The equations are as follows:

(24) $$\begin{array}{c} \mathrm{Acc}=\frac{\mathrm{TP}+\mathrm{TN}}{\mathrm{TP}+\mathrm{TN}+\mathrm{FP}+\mathrm{FN}}, \end{array}$$

(25) $$\begin{array}{c} \text{Sen}=\frac{\mathrm{TP}}{\mathrm{TP}+\mathrm{FN}}, \end{array}$$

(26) $$\begin{array}{c} \mathrm{Spe}=\frac{\mathrm{TN}}{\mathrm{TN+FP}}. \end{array}$$

where Acc, Sen, and Spe represent the accuracy, sensitivity, and specificity, respectively; TP refers to the number of positive samples correctly classified; TN represents the number of negative samples correctly classified; FP represents the negative samples incorrectly classified; and FN indicates the number of positive samples that were misclassified. In practice, the accuracy and recall rates of different scenarios have to be measured:

(27) $$\begin{array}{c} \mathrm{Pre}=\frac{\mathrm{TP}}{\mathrm{FP}+\mathrm{TP}}, \end{array}$$

(28) $$\begin{array}{c} \mathrm{Rec}=\frac{\mathrm{TP}}{\mathrm{FN}+\mathrm{TP}}. \end{array}$$

Then, the *F*1 score can be expressed as

(29) $$\begin{array}{c} F1=2\times \frac{\mathrm{Pre}\times \mathrm{Rec}}{\mathrm{Pre}+\mathrm{Rec}}. \end{array}$$

wherePre represents the precision rate, and Rec refers to the recall rate. The *F*1 score is a weighted average of the model precision rate and the recall rate, and its value range is 0∼1.

### 2.6. Statistical Analysis

In this study, the data were processed using SPSS 19.0 software, and measurement data were expressed as mean ± standard deviation. The classification data were expressed by comparison test, and the data comparison between groups was made by SNK-q test. The parameter correlation was analyzed by Pearson, and *P* < 0.05 indicated the difference was statistically significant.

## 3. Experimental Results

### 3.1. Subjective Evaluation of the Noise Reduction Effect of Different Noise Reduction Algorithms

The 95 patients with suspected fatty degeneration of uterine fibroids who participated in this study were diagnosed with color Doppler ultrasound. The results of the undenatured two-dimensional ultrasound diagnosis are shown in Figure 2. The results showed that the two-dimensional ultrasound of uterine fibroid without degeneration showed an enlarged uterus, smaller fibroids, and a small number. The uterine morphology of most patients was normal. In some patients, the uterine morphology changed due to the effect of fibroids. The echo of the uterine wall was uneven. The submucosal fibroids were separated from the uterine cavity, and the boundary with the endometrium was clear. The internal cervix was opened. The subserosal uterine fibroid could be seen protruding from the surface of the uterus, and the tumors only covered the serosal layer of the uterus. The red color in Figure 2 indicates that the small blood vessels in the fibroids have degenerated and formed thrombi, the hemoglobin has penetrated into the fibroids, and the cut surface is dark red. The acute development of hyalinosis of uterine fibroids, myocyte liquefaction, can be seen in the cystic area staining as light blue cloudy, small clusters of muscle cells remained around the degenerated muscle cells, and there was myocyte proliferation.

The results of ultrasound diagnosis of fatty degeneration of uterine fibroids are shown in Figure 3. The results showed that the patient with fatty degeneration of uterine fibroids showed strong echoes of the tumor in the two-dimensional ultrasound image, the boundary of the muscle wall was obvious and blurred, and there was no attenuation behind. The color blood flow signal was reduced in patients, the high impedance state was obvious, and the surface of uterine fibroids was not covered by the envelope. The circular or semicircular color blood flow signal surrounding the fibroids can be seen around the tumor, some of them could penetrate deep into the fibroids in the star-shaped or short-striped form; and some large fibroids could dilate parauterine blood vessels, which in turn led to increased blood flow. The visual effect suggested that the different noise reduction algorithms in the 3 had a certain inhibitory effect on the noise of the ultrasound image of the patient, but the improved NLM algorithm used in this study was visually superior to the PM algorithm and NLM algorithm. In terms of smoothness, detail retention, and the accuracy of detail judgment, the improved NLM algorithm showed better noise reduction effects on ultrasound images of patients than the PM algorithm and the NLM algorithm. In Figure 3, red indicates scattered small round cells in the fibroids, which can be seen under the microscope, and small vacuoles in the cytoplasm. When the number of lipid droplets was large, they would gather into pieces, showing yellow areas. The vacuoles in the cytoplasm shown in blue were distinguished by special staining.

### 3.2. Objective Evaluation of the Noise Reduction Effects of Different Noise Reduction Algorithms

The noise reduction effects of different noise reduction algorithms on ultrasound images of uterine fibroids patients were evaluated objectively by taking PSNR, MSE, CNR, FOM, and SSIM as the evaluation indicators. The data results of each algorithm after the ultrasound image processing of uterine fibroids patients could be obtained by related calculation. PSNR referred to the ratio between useful signal power and noise power in the image. PSNR was inversely proportional to the degree of image distortion. The larger the PSNR, the smaller the image distortion. The PSNR value of the image after noise reduction based on different algorithms is shown in Figure 4(a). The results of this study showed that the PSNR value of the image before noise reduction was 5.338 dB. After the noise reduction of different algorithms, the PSNR values of all the noise reduction images were greatly improved, which were observably different from those of the original image (*P* < 0.05). The comparison revealed that the optimized NLM algorithm showed a higher PSNR value, which was greatly different from the other two algorithms (*P* < 0.05), suggesting that the improved NLM algorithm had less image distortion after noise reduction.

MSE reflected the degree of gray scale change between the denoised image and the ideal noise-free image. The smaller the image MSE value, the closer the image after noise reduction was to the ideal noise-free image. The MSE value of the image after noise reduction based on different algorithms is shown in Figure 4(b). It indicated that the MSE value of the image before noise reduction was 0.0112. After the noise reduction of different algorithms, the MSE values of all the noise reduction images were improved visibly, showing a statistically significant difference compared with the original image (*P* < 0.05). Compared with the other two algorithms, the improved HLM algorithm showed a smaller MSE value, which indicated that the image processed by the improved HLM algorithm was closer to the ideal image without noise.

CNR referred to the ratio of the difference between the signal intensity and the standard deviations of the background noise of two tissues. It described the processing effect of the noise reduction algorithm on the image. The larger the CNR, the better the processing result. The CNR value of the image after noise reduction based on different algorithms is shown in Figure 4(c). The results of this study showed that the CNR value of the image before noise reduction was 19.38. After noise reduction by different algorithms, the CNR value of all noise-reduced images was several times that of the original image, which was dramatically different from the CNR value of the original image (*P* < 0.05). However, the CNR value of the image after noise reduction using the improved NLM algorithm was much higher than those of the NLM algorithm and the PM algorithm, showing statistically significant differences (*P* < 0.05). Such results suggested that the improved CNR algorithm shows better image contrast.

FOM reflected the effect of the algorithm on image edge keeping. The larger the FOM, the better the edge-keeping effect of the algorithm. As shown in Figure 4(d), the FOM of the ultrasound image before noise reduction was 0.5255, and the FOM value was remarkably increased after the noise reduction processing of different noise reduction algorithms, which was significantly different from that of the original image (*P* < 0.05). On this basis, the improved NLM algorithm proposed in this study showed a higher FOM value, indicating that the improved NLM algorithm could better improve the edge-keeping effect of the ultrasound image without affecting the image noise reduction effect.

SSIM was to show the structural integrity of the noise-reduced image, and it could evaluate the image quality by comparing the changes in image brightness, contrast, and structure. Figure 4(e) illustrates the PSNR values of the image after noise reduction based on different algorithms. The SSIM value of the ultrasound image before noise reduction was 0.4231. It was reduced obviously after noise reduction by different algorithms, showing an observable difference in contrast to the original image (*P* < 0.05). However, the SSIM value of the improved NLM algorithm was significantly higher in contrast to the NLM algorithm and the PM algorithm after noise reduction, and the differences were statistically significant (*P* < 0.05), suggesting that the improved NLM algorithm showed less image distortion and more image structure after the noise reduction.

### 3.3. Comparison of Image Noise Reduction Times Based on Different Algorithms

The running time of different algorithms was counted when noise reduction was performed on ultrasound images of uterine fibroids patients (Figure 5). The results showed that the average noise reduction time of the PM algorithm, the NLM algorithm, and the improved NLM algorithm was 16.38 ± 4.33 s, 18.01 ± 5.14 s, and 23.81 ± 4.62 s, respectively. Although the improved NLM algorithm greatly improved the diagnostic effect of fatty degeneration of uterine fibroids, the noise reduction time of the algorithm was slightly longer.

### 3.4. Ultrasound Diagnosis Results of Uterine Fibroids Patients Based on Different Noise Reduction Algorithms

In this study, 95 patients with suspected fatty degeneration of uterine fibroids were diagnosed by surgery and pathology, and 64 patients were confirmed as fatty degeneration, including 46 patients with fatty degeneration of intramural fibroids, 15 patients with fatty degeneration of subserosal fibroids, and 5 cases of fatty degeneration of submucosal fibroids. Diagnosis results (as illustrated in Figures 6–9) based on different ultrasonic imaging noise reduction algorithms revealed that before the noise reduction of the image, there were 38 cases of intramural fibroids (8 cases with missed diagnosis), 10 cases of fatty degeneration of subserosal fibroids (5 cases with missed diagnosis), and 2 cases of fatty degeneration of submucosal fibroids (3 cases with missed diagnosis). After noise reduction using the PM algorithm, 40 cases were diagnosed with fatty degeneration of intermural fibroids (6 cases with missed diagnosis), 11 cases of fatty degeneration of subserosal fibroids (4 patients with missed diagnoses), and 2 cases of fatty degeneration of submucosal fibroids (3 cases of missed diagnosis). After noise reduction using the NLM algorithm, 43 cases were diagnosed with fatty degeneration of intramural fibroids (3 cases of missed diagnosis), 12 cases were confirmed as fatty degeneration of subserosal fibroids (3 cases of missed diagnosis), and there were 2 patients with fatty degeneration of submucosal fibroids (3 cases of missed diagnosis). After noise reduction using the improved NLM algorithm, the images showed that there are 46 cases with fatty degeneration of intermural fibroids, 15 cases with fatty degeneration of subserosal fibroids, and 4 cases of fatty degeneration of submucosal fibroids, with 1 case of missed diagnosis. The diagnosis rate before improvement was 75.0%, PM diagnosis accuracy rate was 79.69%, and NLM algorithm diagnosis rate was 85.94%. Comparison indicated that the diagnosis results of the algorithm proposed in this study were closer to the pathological diagnosis results, showing no statistically significant difference (*P* > 0.05). Such results suggested that the improved NLM algorithm showed a more obvious diagnosis effect after noise reduction of the ultrasound image of the patient.

## 4. Discussion

Uterine fibroid is a disease in which uterine smooth muscle cells are proliferated due to s [22]. Excessive body fat deposition leads to gynecological diseases, symptoms such as irregular menstruation, bloated body, and inconvenient movement, which increase the probability of uterine fibroids. There is a certain relationship between body fat deposition and uterine fibroids [23]. Ultrasound examination of uterine fibroids should pay attention to the differentiation of endometrial lesions and uterine sarcomas. Ultrasound examination of uterine fibroids and sarcomas can manifest as heterogeneous plaque-like hyperechoic similar to fatty changes of fibroids. Color Doppler ultrasound is more conducive to diagnosis. Some scholars use magnetic resonance imaging to quantitatively differentiate the fat deposition of human organs and tissues to improve the reliability of fat scores [24]. There is no envelope for uterine fibroids, and their blood vessel walls lack outer membrane protection, which can easily cause fibroids blood supply disorder when compressed and lead to various degenerations. Common uterine fibroid degeneration includes hyalinosis, mucus degeneration, red degeneration, steatosis, calcification, and cystic degeneration. Even sarcomatoid degeneration may be caused in severe cases [25, 26]. Fatty degeneration accounts for only about 0.2% of the degeneration of uterine fibroids. Most fatty degeneration of uterine fibroids occurs after hyaline degeneration or necrosis. The degeneration lesions are usually small and difficult to distinguish or detect by the naked eye, and yellow dots can be seen only. Therefore, it is easy to be misdiagnosed as lipoma [27]. Ultrasound is the preferred method for clinical examination of uterine fibroids. Undenatured uterine fibroids and steatotic uterine fibroids show different imaging morphologies under ultrasound. Therefore, ultrasound diagnosis of fatty degeneration of uterine fibroids has a significant value. Sun et al. [17] provided a diagnostic algorithm based on magnetic resonance imaging, which considered morphological and functional characteristics, including single and combined, to optimize the radiological discrimination between leiomyomas and leiomyosarcomas. High-intensity focused ultrasound therapy has received more and more attention in treating benign uterine tumors. Magnetic resonance or ultrasound imaging has been used to target and monitor the ablation process. Cheung et al. [28] outlined the background, clinical application, treatment results, and safety of high-intensity focused ultrasound in treating uterine fibroids and adenomyosis, including clinical trial summaries that compare high-intensity focused ultrasound guided by magnetic resonance or ultrasound with other minimally invasive or surgical interventions. This treatment can retain the uterus as another option for women with uterine fibroids and adenomyosis. Lee et al. [29] proved that ultrasound-guided high-intensity focused ultrasound (USgHIFU) ablation was effective in treating uterine fibroids and adenomyosis and did not affect ovarian reserve.

Based on the traditional NLM algorithm, this study improves the Euclidean distance from the three aspects of the block median, the block average, and the gray value of the central pixel of the two pixel blocks and uses ultrasound to detect the fat deformation of uterine fibroids. In addition, the gradient value of the NLM algorithm in the calculation process was reduced, and the overall algorithm was adjusted using the cosine function to improve the noise reduction effect of the NLM algorithm. After the noise reduction effects based on different noise reduction algorithms were evaluated, it was found that the improved NLM algorithm was much better than the PM algorithm and the NLM algorithm in terms of smoothness, detail preservation, and detail judgment on the patient's ultrasound image. The objective evaluation revealed that after the noise reduction by using improved NLM algorithm on the ultrasound images of uterine fibroids patients, the PSNR, CNR, FOM, and SSIM were significantly higher in contrast to those of the PM algorithm and the NLM algorithm, and the differences were statistically significant (*P* < 0.05). The MSE after the noise reduction by the improved NLM algorithm was much lower than the PM algorithm and the NLM algorithm, showing a statistically significant difference (*P* < 0.05). Based on the above five indicators, the improved NLM algorithm had significantly better image noise reduction effects than the other two algorithms. However, the improved NLM algorithm reduced the noise a little longer from the point of view of noise reduction time. Diagnosis of fatty degeneration of uterine fibroids showed that after the ultrasound images were processed by the NLM algorithm to reduce noise, there were 46 cases of intermural fibroids, 15 cases of subserosal fibroids, and 4 cases of submucosal fibroids. Only one case with submucosal fibroids steatosis was missed diagnosis, showing no significant difference in contrast to the pathological examination results (*P* > 0.05). Compared with the diagnosis results based on the PM algorithm and the NLM algorithm, the improved NLM algorithm significantly improved the diagnosis accuracy of the fatty degeneration of uterine fibroids.

## 5. Conclusion

The NLM algorithm was improved by changing the gradient of the traditional algorithm and introducing the cosine function. It was applied to the ultrasonic imaging intelligent diagnosis of fatty degeneration of uterine fibroids patients in this study. The diagnosis rate before improvement was 75.0%, the diagnosis accuracy rate for PM was 79.69%, and the diagnosis rate after improvement was 85.94%.

The improved NLM algorithm had a good noise reduction effect on ultrasound images of patients with uterine fibroids. However, there were still some shortcomings in this study. The algorithm had not analyzed the auxiliary effect of the algorithm in treating patients with fatty degeneration of uterine fibroids. Therefore, there was a lack of guiding significance for the clinical auxiliary treatment of patients with fatty degeneration of uterine fibroids, which had to be confirmed by more clinical studies. Ultrasound images with intelligent noise reduction algorithms are worth popularizing clinically for evaluating steatosis of uterine fibroids.

## Figures and Tables

**Figure 1:** Calculating process of improved NLM algorithm.

**Figure 2:** The noise reduction effect of different noise reduction algorithms on ultrasound images of patients with uterine fibroids. (a) The noise reduction effect of the improved NLM algorithm. (b) The noise reduction effect of the NLM algorithm. (c) The noise reduction effect of the PM algorithm. (d) The noise-reduced image.

**Figure 3:** The noise reduction effects of different noise reduction algorithms on ultrasound images of fatty degeneration of uterine fibroids. (a, b, c) Noise reduction effects of the improved NLM algorithm, NLM algorithm, PM algorithm, respectively; and (d) the noise-reduced image.

**Figure 4:** The objective evaluation results of different noise reduction algorithms on the noise reduction effect of ultrasound images of uterine fibroids patients. ^*∗*^indicates that the difference was statistically obvious (*P* < 0.05).

**Figure 5:** Comparison of running time based on different noise reduction algorithms. ^*∗*^indicates that the difference was statistically obvious (*P* < 0.05).

**Figure 6:** Diagnosis results of different algorithms for fatty degeneration of intermural fibroids. ^*∗*^indicates that the difference was statistically significant (*P* < 0.05).

**Figure 7:** Diagnosis results of different algorithms for fatty degeneration of subserosal fibroids. ^*∗*^indicates that the difference was statistically significant (*P* < 0.05).

**Figure 8:** Diagnosis results of different algorithms for fatty degeneration of submucosal fibroids. ^*∗*^indicates that the difference was statistically significant (*P* < 0.05).

**Figure 9:** Diagnosis results of different algorithms for fatty degeneration of uterine fibroids. ^*∗*^indicates that the difference was statistically significant (*P* < 0.05).

## Data Availability

The data used to support the findings of this study are available from the corresponding author upon request.
